The article "Comparison of Steroid-Free Immunosuppression and Standard Immunosuppression for Liver Transplant Patients with Hepatocellular Carcinoma" was retracted in 2019. Reasons: lack of ethics approval or compliance; missing or withdrawn patient consent; ethical violations by an author; concerns about the data.

# Comparison of Steroid-Free Immunosuppression and Standard Immunosuppression for Liver Transplant Patients with Hepatocellular Carcinoma

**DOI:** 10.1371/journal.pone.0071251

**Published:** 2013-08-06

**Authors:** Tonghai Xing, Li Huang, Zhenhai Yu, Lin Zhong, Shuyun Wang, Zhihai Peng

**Affiliations:** 1 Department of General Surgery, Shanghai First People’s Hospital, Shanghai Jiao Tong University, Organ Transplantation Center of Shanghai, Shanghai, China; 2 Department of General Surgery, Shandong Qianfoshan Hospital, Ji’nan, China; St. Luc University Hospital, Belgium

## Abstract

Immunosuppression therapy following liver transplantation often includes steroids. However, extended corticosteroid therapy is associated with numerous complications. This study evaluated the efficacy and safety of using basiliximab in place of a corticosteroid for immunosuppression following liver transplantation for hepatocellular carcinoma (HCC) in Chinese patients. The records of 178 patients with HCC who underwent orthotopic liver transplantation from January 2003 to December 2009 were retrospectively reviewed. All patients received immunosuppression therapy that contained either basiliximab (n = 78) or steroids (n = 100) in addition to tacrolimus and mycophenolate mofetil. Assessments included complications related to liver transplantation, occurrence of steroid side effects, recurrence of HCC, and patient and graft survival. A smaller proportion of patients receiving basiliximab compared with steroids experienced *de novo* diabetes (38.7% vs. 91.0%, respectively) or long-term *de novo* diabetes mellitus (7.7% vs. 38.0%, respectively) (both, *P*<0.0001). The median overall and disease free survival was similar between basiliximab (50.8 months and 19.6 months, respectively) and steroid treated patients (64.2 months and 23.8 months, respectively). The 5-year overall survival and disease free survival rates was also similar between the basiliximab (42.5% and 38.9%, respectively) and steroid (50.5% and 39.2%) groups (all, *P*>0.730). However, in patients who met the Milan criteria basiliximab was associated with greater 5-year overall survival rate as compared with steroid therapy (88.9% vs. 57.4%, respectively, *P = *0.022). These findings provide further evidence of the negative impact of steroids as a part of immunosuppression therapy following liver transplantation for HCC.

## Introduction

Hepatocellular carcinoma (HCC) is the third most frequent cause of cancer death worldwide [1]. In 2008, it was estimated that about 700,000 cancer deaths were due to HCC, and half of these were in China [1]. Major risk factors for HCC include chronic infections with hepatitis B (HBV) or C (HCV) viruses, foodstuff contamination with aflatoxins, and increased alcohol consumption [2]–[5]. Approximately 7% of the population in China are positive for HBV, and the elevated presence of HBV infection is reflected in the higher rate of HCC in China [6], [7].

Orthotopic liver transplantation (OLT) is the treatment of choice for patients with hepatic cirrhosis related to HCC [8]. Standard immunosuppressive treatment following liver transplantation includes corticosteroids and calcineurin inhibitors (CNIs). This treatment strategy has improved survival of patients with liver transplants; however, long-term steroid-based immunosuppression is associated with serious complications and increased morbidity and mortality [9]. Existing evidence suggests that extended corticosteroid therapy is associated with complications including diabetes, hypercholesterolemia, and atrial hypertension [9], [10].

Recent treatment strategies have been aimed at limiting corticosteroid use to improve the quality of life in transplant recipients [11]. Promising clinical results with the CNI tacrolimus in liver transplant patients have resulted in the development of tacrolimus-based protocols with minimal use of corticosteroids [11]–[14].

Basiliximab is a monoclonal antibody to the α chain of the interleukin (IL)-2 receptor of T-cells, and is used to prevent organ rejection following transplantation [15]. Several studies have investigated the use of basiliximab as part of immunosuppression therapy in liver transplant recipients [16]–[20], but only a few have examined its use the absence of steroids [16], [19]. Prior studies have found that the choice of immunosuppressive therapy can affect outcomes, including recurrence of HCC [21], [22]. The objective of this study was to compare the clinical outcomes of Chinese HCC patients who received basiliximab as part of their immunosuppressive therapy with those who received steroid-based therapy following liver transplantation.

## Methods

This study was a retrospective chart review of patients who underwent OLT at the Department of General Surgery, Shanghai First People’s Hospital between January 2003 and December 2009. The study was approved by the ethics committee of the hospital, and followed the principles of the Declaration of Helsinki. Written consent was given by the patients for their information to be stored in the hospital database and used for research.

### Study Population

Eligible patients were ≥ 18 years or age and had undergone cadaveric OLT for histologically proven HCC. The criteria for a patient being eligible for liver transplantation in China differ from those used in Western countries. In China, there are 2 criteria, the Hangzhou and Shanghai criteria. The Hangzhou criterion specify a total tumor diameter ≤8 cm, or a total tumor diameter >8 cm with a histopathological grade I or II, and preoperative alpha-fetoprotein level ≤400 ng/mL. The Shanghai criterion requires a solitary lesion ≤9 cm without macrovascular or lymph node invasion, or extrahepatic metastasis [23], [24]. Patients were not included in this study if they received a liver transplant for acute liver failure, received multiple organ transplantation, had received more than one liver transplant, had prior transplants of other organs, had autoimmune hepatitis, biliary cirrhosis, ABO-ABO-incompatible liver transplantation, or were infected with human immunodeficiency virus.

### Study Design

Medical records were reviewed for demographic and pre-, intra- and post-operative clinical information. Patients were retrospectively classified by the traditional Milan criteria (single tumor ≤5 cm, or 2–3 tumors with none exceeding 3 cm, and no vascular invasion and/or extrahepatic spread) [21] and the University of California San Francisco (UCSF) criteria (single tumor ≤6.5 cm, or 2–3 tumors with none exceeding 4.5 cm with a total tumor diameter ≤8 cm, and no vascular invasion and/or extrahepatic spread) [22]. All patients received methylprednisolone 500 mg as a single intravenous dose before reperfusion during the transplantation procedure. Patients who received steroid-based immunosuppressive induction therapy also received intravenous methylprednisolone on days 1 through 7 after transplantation, beginning at 300 mg/day on day 1 and tapering down to 40 mg/day on day 7. These patients subsequently received oral prednisone from day 8 through day 90, beginning at 20 mg/day on day 8, and followed a gradual tapering schedule to discontinuation.

Patients not receiving steroid-based therapy post-operatively received 2 doses of intravenous basiliximab 20 mg, with the first dose at 6 hours after reperfusion and a second dose on postoperative day 4.

Postoperatively, all patients received the CNI inhibitor tacrolimus in combination with mycophenolate mofetil (MMF). Tacrolimus was initiated at an oral dose of 0.05 mg/kg/day in two divided doses. The dose was subsequently adjusted to achieve a whole blood trough concentration (measured just prior to the next dose) of 5–10 ng/mL. Tacrolimus treatment was withheld when patients showed insufficient renal function (creatinine >120 µmol/L or creatinine clearance <40 mL/min). MMF, 750 mg twice daily, was initiated after confirmation of the absence of pancytopenia (hematocrit >26% and platelet count >50,000 cells/mm^3^). At 90 days post-surgery, immunosuppressive therapy was steroid-free for all patients. If there was mild to moderate rejection of the transplanted liver, the dose of tacrolimus or MMF was increased. If there was severe rejection, patients were given methylprednisolone (500 mg) for 3 days with or without an increase in tacrolimus or MMF.

All acute rejection episodes were verified by liver biopsy, and if confirmed using the criteria of the fifth Banff Consensus conference [23], patients received an intravenous bolus of 500 mg methylprednisolone per day for 3 consecutive days. If liver function tests showed improvement, steroid therapy with oral methylprednisolone or prednisone was continued. If liver function did not improve, the rejection episode was considered to be steroid-resistant and the tacrolimus dose was increased (0.1 mg/kg/day in two divided doses to achieve 8–10 ng/mL whole blood trough concentration levels) and no steroids were given. The dose of MMF could be increased as determined by the treating physician.

Anti-infective prophylaxis was administered according to local practice. The most common protocol was the administration of antibiotics (amoxicillin/clavulanate or aztreonam) for 5 to 7 days without antiviral prophylaxis. Antiviral prophylaxis with valganciclovir was administered only to cytomegalovirus (CMV) mismatch patients (CMV IgG-positive donor/CMV IgG-negative recipient). The postoperative anti-HBV protocol included administration of lamivudine plus low-dose intramuscular HBV immunoglobulin [24].

All patients were followed-up in outpatient clinics until of the end of 2012.

### Study Assessments

The primary endpoints were patient overall survival (OS) and disease-free survival (DFS). Secondary endpoints included the incidence of biopsy-proven acute rejection, the incidence and severity of HCC recurrence, graft survival, recurrence of HBV infection, incidence of adverse events related to immunosuppressive therapy, incidence of infection, and incidence of metabolic complications (diabetes mellitus, hypertension, and hyperlipidemia).

Diabetes mellitus, hypertension, and hyperlipidemia were diagnosed according to the guidelines of the World Health Organization. *De novo* diabetes was defined as diabetes mellitus diagnosed within 30 days postoperatively in patients who did not have diabetes before transplantation. Long-term *de novo* diabetes was defined as diabetes mellitus newly diagnosed within 30 days postoperatively with active disease continuing beyond 30 days postoperatively. *De novo* hypertension and *de novo* hyperlipidemia were defined as hypertension and hyperlipidemia newly diagnosed within one year postoperatively in patients who did not have these conditions preoperatively.

Recurrence of HCC was monitored by ultrasonography performed monthly for 6 months, and then every 3 months for the first year, every 6 months for the second year, then annually thereafter. Computed tomography (CT) scans were performed if the results of the ultrasonography were not conclusive. HCC recurrence was also monitored by measurement of alpha fetoprotein serum levels every month for 6 months, followed by every 2 months for the next 6 months, then biannually.

Recurrence of HBV was monitored by evaluating presence of HBV surface antigen and HBV DNA in serum. These tests were performed at each follow up visit.

Biopsies were performed when clinically required.

Patients were evaluated for these outcomes during their postoperative hospital stay, and their follow-up examinations at 1, 2, 3, 6, 9, and 12 months during the first year post-surgery, and every 3–6 months in subsequent years.

### Statistical Analysis

Continuous variables were summarized by mean ± standard deviation or median with inter-quartile range (IQR, the range between the 25^th^ and 75^th^ percentile) depending on normality of the distribution of the data. Categorical variables were expressed by frequencies and percentages. The differences in the distribution of the demographic and clinical characteristics between the steroid and basiliximab groups were detected by independent t-test or Wilcoxon rank sum test for continuous variables, and by Chi-square test or Fisher’s exact test for categorical variables, as appropriate.

Overall survival (OS) time was defined as the length of time from the date of liver transplantation to the date of death or last follow up visit. Patients were censored in the DFS analysis if they were disease free (without HCC recurrence) at the last visit, but either HCC recurrence or death was counted as an event in the DFS analysis. The survival curves were constructed by the Kaplan-Meier method with log-rank test to detect the difference between the basiliximab and steroid groups, for OS and DFS, respectively. Kaplan-Meier survival curves for DFS were also constructed for patients based on the Milan and UCSF criteria.

Cox’s proportional hazard regressions were performed to calculate crude and adjusted hazard ratios (HRs), with 95% confidence interval (CIs), for effects of immunosuppression therapy group (basiliximab vs. steroid group) and other potential prognostic factors of OS and DFS. The multivariate Cox’s proportional hazard regression model was constructed using the backward selection procedure, wherein variables that did not improve the model fit at *P*<0.05 were discarded. Treatment group, age, gender, and transplant year were always forced in the model for adjustment. The statistical analyses were all performed with SAS software version 9.2 (SAS Institute Inc., Cary, North Carolina). A two-tailed *P*<0.05 indicated statistical significance.

## Results

### Recipient Demographic and Baseline Characteristics

Of the 543 patients who received a liver transplant at our hospital, 178 were eligible for the study (Figure 1). There were more males (n = 156 [87.6%]) than females (n = 22 [12.4%], and the mean age of the patients was 49.2±8.7 years (range, 21.3 to 72.9 years). The distribution of age, gender, alpha-fetoprotein level, Child-Pugh score, type of HCC, meeting of the Milan and UCSF criteria, presence of diabetes mellitus, hypertension, hyperlipidemia, HBV infection, HCV infection, cirrhosis, and treatment with preoperative antiviral therapy were similar between the basiliximab and steroid group (all *P*>0.05; Table 1). Tumor number, size, and stage were similar between groups (Table 1). The distribution of transplant year was significantly different between the two groups (*P*<0.0001); all patients who received a liver transplant prior to 2006 were given steroid therapy, and most patients from 2007 to 2009 received basiliximab therapy (Table 1).

**Figure 1:** Consort diagram.

**Table 1:** Recipient demographic and pre-operative characteristics.

	Basiliximab (n = 78)	Steroid (n = 100)	*P*-value
Gender			
Female	7 (9.0)	15 (15.0)	0.226¶
Male	71 (91.0)	85 (85.0)	
Age	48.7±8.4	49.6±8.9	0.485†
AFP^1^	207.0 (6.3, 897.3)	200.0 (24.5, 1000.0)	0.497‡
Transplant year			
2003–2005	0 (0.0)	79 (79.0)	<0.0001¶
2006–2009	78 (1.00)	21 (21.0)	
Child–Pugh score^2^			
5–6	40 (52.0)	46 (46.0)	0.211¶
7–9	33 (42.9)	41 (41.0)	
10–15	4 (5.2)	13 (13.0)	
HCC			
Primary cancer	69 (88.5)	93 (93.0)	0.294¶
Recurrent cancer	9 (11.5)	7 (7.0)	
HBV positive	72 (92.3)	92 (92.0)	0.940¶
HCV positive	1 (1.3)	2 (2.0)	1.000§
Cirrhosis	68 (87.2)	93 (93.0)	0.190¶
Number of tumors	1.0 (1.0, 4.0)	1.0 (1.0, 3.0)	0.247†
Diameter of largest tumor (cm)	3.8 (2.0, 7.0)	4.0 (2.2, 8.5)	0.479†
TNM tumor stage			
Stage I	15 (19.2)	26 (26.0)	0.135¶
Stage II	23 (29.5)	38 (38.0)	
Stage III	39 (50.0)	36 (36.0)	
Stage IV	1 (1.3)	0 (0.0)	
Milan Criteria^2^			
Within Milan	28 (36.4)	36 (36.0)	0.960¶
Beyond Milan	49 (63.6)	64 (64.0)	
UCSF Criteria^1^			
Within UCSF	31 (40.8)	40 (41.2)	0.953¶
Beyond UCSF	45 (59.2)	57 (58.8)	
Diabetes mellitus	3 (3.9)	11 (11.0)	0.079¶
Hypertension	6 (7.7)	6 (6.0)	0.655¶
Hyperlipidemia	3 (3.8)	0 (0.0)	0.082§
Preoperative antiviral therapy	16 (20.5)	30 (30.0)	0.151¶

Data are presented as number (percentage), median (IRQ), or mean ± standard deviation.

† Independent t-test;

‡ Wilcoxon rank sum test;

¶ Chi-square test;

§ Fisher’s exact test.

1 Two subjects in basiliximab group and three in the steroid group were missing data.

2 One subject in basiliximab group was missing data.

AFP = alpha-fetoprotein; HBV = hepatitis B virus; HCC = hepatocellular carcinoma; HCV = hepatitis C virus; IQR = interquartile range; SD, standard deviation; UCSF, University of California San Francisco.

### Recipient Postoperative Status, Complications, Steroid Side Effects, and Postoperative Immunosuppression

Following liver transplantation, the median follow-up time in the basiliximab and steroid groups was 37.2 (8.7, 52.6) months and 19.5 (4.1, 83.3) months, respectively (*P* = 0.819), and the mean follow-up time in the two groups was 33.4±23.8 months and 39.9±40.1 months, respectively (*P* = 0.180) (Table 2). In both treatment groups, most patients did not experience recurrence of HBV (>88%) (*P* = 0.099) or *de novo* HBV infection (>66%) (*P* = 1.0).

**Table 2:** Recipient postoperative status, complications, and immunosuppressive therapy^a^.

		Basiliximab (n = 78)		Steroid (n = 100)	*P*-value
Follow-up time (month)					
Median (IQR)		37.2 (8.7, 52.6)		19.5 (4.1, 83.3)	0.819†
Mean ± SD		33.4±23.8		39.9±40.1	0.180§
Mortality, perioperative period		4 (5.1)		11 (11.0)	0.162‡
Mortality		34 (43.6)		42 (42.0)	0.832‡
Cause of death					
Graft failure		1 (2.9)		1 (2.4)	0.591‡
Hemorrhage		3 (8.8)		1 (2.4)	
Multi-organ failure		22 (64.7)		30 (71.4)	
Respiratory complication		1 (2.9)		1 (2.4)	
Died after re-transplantation		1 (2.9)		4 (9.5)	
Recurrent disease		6 (17.7)		4 (9.5)	
Other		0 (0.0)		1 (2.4)	
HBV recurrence	n = 72	8 (11.1)	n = 92	4 (4.4)	0.099‡
*De novo* HBV infection	n = 6	2 (33.3)	n = 8	2 (25.0)	1.000¶
*De novo* diabetes	n = 75	29 (38.7)	n = 89	81 (91.0)	<0.0001‡
Long-term *de novo* diabetes	n = 75	3 (4.0)	n = 89	27 (30.3)	<0.0001‡
*De novo* hypertension	n = 72	4 (5.6)	n = 94	5 (5.3)	1.000¶
*De novo* hyperlipidemia	n = 75	3 (4.0)		1 (1.0)	0.315¶
Pleural effusion		63 (80.8)		54 (54.0)	0.0002‡
Postoperative infection		33 (42.3)		23 (23.0)	0.006‡
Biliary complication		6 (7.7)		5 (5.0)	0.538¶
Renal failure		1 (1.3)		7 (7.0)	0.081¶
Pulmonary edema		2 (2.6)		5 (5.0)	0.469
Intra-abdominal bleeding		7 (9.0)		5 (5.0)	0.294‡
Intra-abdominal collection/abscess		6 (7.7)		1 (1.0)	0.045¶
Vascular complication		2 (2.6)		3 (3.0)	1.000¶
CMVpp65 antigenemia		0 (0.0)		1 (1.0)	1.000¶
Primary graft nonfunction		0 (0.0)		1 (1.0)	1.000¶
Chronic rejection		0 (0.0)		0 (0.0)	NA
GVHD		0 (0.0)		0 (0.0)	NA
PTLD		0 (0.0)		0 (0.0)	NA
***Postoperative immunosuppressive therapy*** b					
Recipient alive at end of study		44 (56.4)		58 (58.0)	
Maintenance immunosuppressant					
Tacrolimus		42 (95.5)		54 (93.1)	0.697¶
MMF		40 (90.9)		58 (100.0)	0.032¶
Sirolimus		0 (0.0)		5 (8.6)	0.068¶
Immunosuppression protocol, n (%)					
Tacrolimus+MMF+sirolimus		0 (0.0)		5 (8.6)	0.017¶
Tacrolimus+MMF		38 (86.4)		49 (84.5)	
Tacrolimus only		4 (9.1)		0 (0.0)	
MMF only		2 (4.6)		4 (6.9)	

Data are presented as number (percentage), median (IRQ), or mean ± standard deviation.

a The number of patients for the basiliximab and steroid groups are 78 and 100, respectively unless indicated otherwise.

b The number of patients for the basiliximab and steroid groups are 44 and 58, respectively.

† Wilcoxon rank sum test;

‡ Chi-square test;

¶ Fisher’s exact test;

§ independent t-test.

CMV = cytomegalovirus; GVHD = graft versus host disease; MMF = mycophenolate mofetil; NA = not available; PTLD = post-transplant lymphoproliferative disorder.

Table 2 summarizes the postoperative complications and steroid side effects. A lower proportion of patients treated with basiliximab compared with steroids had *de novo* diabetes and long-term *de novo* diabetes (both, *P*<0.0001). A greater percentage of basiliximab patients experienced pleural effusion, postoperative infection, and intra-abdominal collection/abscess compared with those treated with steroids (all, *P*<0.05). Other complications were comparable between the two groups. No patients experienced chronic rejection, graft versus host disease (GVHD), or post-transplant lymphoproliferative disorder (PTLD).

Of the surviving patients at the end of the study who received immunosuppression therapy, more patients in the steroid group required MMF as compared to the basiliximab group (100.0% vs. 90.9%, respectively; *P* = 0.032) (Table 2). The distribution of immunosuppression protocols between two groups were significantly different (*P* = 0.017), with the most common treatment for both groups being tacrolimus plus MMF (>80%) (Table 2).

Of the surviving patients receiving immunosuppression therapy, one patient in the steroid group and three in the basiliximab group were switched from a CNI to sirolimus due to the occurrence of renal dysfunction as evidenced by elevated creatinine and proteinuria. MMF was discontinued in one patient in the steroid group and three patients in the basiliximab group due to leukopenia (white blood cell count <2000/mm^3^).

### Recipients with Acute Rejection

A total of 22 patients experienced biopsy-proven acute rejection, and the rejection rate was similar between the groups (*P = *0.869) (Table 3). The rejection time was significantly different between basiliximab and steroid treated patients (*P* = 0.013). In the basiliximab group, rejection most often occurred within the first 2 weeks, and in the steroid group between 2 and 6 months (Table 3). All patients had mild to moderate rejection severity based on Banff’s schema for grading liver allograft rejection; no cases of severe rejection occurred. All episodes of rejection were successfully treated. The revised treatments protocols used to treat acute rejection did not differ between the groups (all, *P* = 0.67), and basiliximab and steroid treated patients had similar mortality per revised treatment protocol (Table 3). For both treatment groups, the most common revised protocol was tacrolimus and glucocorticoids.

**Table 3:** Recipients with acute rejection.

	Basiliximab (n = 78)	Steroid (n = 100)	*P*-value
Acute rejection	10 (12.8)	12 (12.0)	0.869†
Rejection time after transplantation			
0–14 days	8 (80.0)	2 (16.7)	0.013‡
15–30 days	2 (20.0)	6 (50.0)	
2–6 months	0 (0.0)	3 (25.0)	
7–12 months	0 (0.0)	1 (8.3)	
Revised treatment protocol			
Tacrolimus	4 (40.0)	4 (33.3)	0.607‡
Glucocorticoid^a^	3 (30.0)	6 (50.0)	
MMF	1 (10.0)	0 (0.0)	
Tacrolimus+glucocorticoid^a^	1 (10.0)	0 (0.0)	
Tacrolimus+MMF	1 (10.0)	2 (16.7)	
Mortality, by revised treatment protocol			
Tacrolimus	1 (25.0)	2 (50.0)	1.000‡
Glucocorticoid^a^	2 (66.7)	4 (66.7)	1.000‡
MMF	0 (0.0)	–	NA
Tacrolimus+glucocorticoid^a^	1 (100.0)	–	NA
Tacrolimus+MMF	0 (0.0)	0 (0.0)	NA

Data are presented as number (percentage).

a Glucocorticoid treatment consisted of oral methylprednisolone or oral prednisone.

† Chi-square test;

‡ Fisher’s exact test.

MMF = mycophenolate mofetil, NA = non-available.

### Recipients with HCC Recurrence

HCC recurred at a similar frequency in patients in the basiliximab and steroid groups (44.9% vs. 38.0%, respectively; *P = *0.355) (Table 4). Approximately one quarter of patients in each group experienced intrahepatic recurrence and extrahepatic recurrence with no statistically significant differences in rates between groups (Table 4). For extrahepatic recurrence, the most common site was the lung (77.3% and 56.5% for basiliximab and steroid patients, respectively). About 40% of patients in both groups experienced HCC recurrence within 1 year, with 28.4% having intrahepatic recurrence and 28.4% have extrahepatic recurrence. None of the three patients positive for HCV experienced HCV recurrence.

**Table 4:** Recipients with HCC Recurrence^a^.

		Basiliximab(n = 78)		Steroid(n = 100)	*P*-value
Overall recurrence of HCC		35 (44.9)		38 (38.0)	0.355†
Intrahepatic recurrence^b^	n = 74	25 (33.8)	n = 94	29 (30.9)	0.686†
Extrahepatic recurrence/transfer^b^	n = 74	23 (31.1)	n = 94	23 (24.5)	0.340†
Transferred location^c^					
Lung	n = 22	17 (77.3)		13 (56.5)	0.458‡
Bone	n = 22	2 (9.1)		4 (17.4)	
Lung+bone	n = 22	2 (9.1)		2 (8.7)	
Bone+brain	n = 22	0 (0.0)		1 (4.4)	
Lung+bone+brain	n = 22	1 (4.6)		0 (0.0)	
Lung+brain	n = 22	0 (0.0)		1 (4.4)	
Abdomen	n = 22	0 (0.0)		2 (8.7)	
Recurrence of HCC within 1 year		29 (37.2)		28 (28.0)	0.193†
Intrahepatic recurrence within 1 year^b^	n = 74	21 (28.4)	n = 94	21 (22.3)	0.370†
Extrahepatic recurrence/transfer within 1 year^b^	n = 74	21 (28.4)	n = 94	18 (19.2)	0.160†
Transferred location within 1 year^c^					
Lung	n = 20	16 (80.0)		9 (50.0)	0.199‡
Bone	n = 20	2 (10.0)		4 (22.2)	
Lung+bone	n = 20	1 (5.0)		2 (11.1)	
Lung+bone+brain	n = 20	1 (5.0)		0 (0.0)	
Lung+brain	n = 20	0 (0.0)		1 (5.6)	
Abdomen	n = 20	0 (0.0)		2 (11.1)	

Data are presented as number (percentage).

a The number of patients for basiliximab and steroid groups are 78 and 100, respectively unless indicated otherwise.

† Chi-square test;

‡ Fisher’s exact test. NA: non-available.

b Four subjects in the basiliximab group and 6 subjects in the steroid group had missing data.

c One subject in the basiliximab group was missing data.

HCC = hepatocellular carcinoma.

### Overall Survival and Disease-free Survival

In the two groups, 5.1% of the patients receiving basiliximab and 11.0% of the patients receiving steroids died within 1 month postoperatively. During the course of the study, a similar number of patients died in the basiliximab (43.6%) and steroid (42.0%) groups (*P* = 0.832). The most common cause of death for the basiliximab and steroid groups was multiple organ failure (64.7% and 71.4%, respectively), and the second most common cause of death was recurrent disease (17.7% and 9.5%, respectively).

The median OS and DFS for the basiliximab group were 50.8 months and 19.6 months, respectively, and for the steroid group were 64.2 months and 23.8 months, respectively. The 5-year OS rate was similar between the basiliximab and steroid groups (42.5% vs. 50.5%; *P = *0.734) (Figure 2), as was the 5-years DFS rate (38.9% vs. 39.2%; *P = *0.913) (Figure 3a).

**Figure 2:** Overall survival of recipients between basiliximab and steroid groups (log-rank test, *P = *0.734).

**Figure 3:** Disease-free survival between basiliximab and steroid groups for (A) all recipients (log-rank test, *P = *0.913); (B) recipients within Milan criteria (log-rank test, *P = *0.022); (C) recipients within UCSF criteria (log-rank test, *P = *0.079).

In the group of patients with HCC exceeding the Milan criteria, there were 64 patients in the steroid group and 50 patients in the basiliximab, and based on follow-up to date there are 12/64 and 11/50 patients who survived in the steroid and basiliximab groups, respectively. Stratifying patients by the Milan and UCSF criteria indicated that the 5-year OS rate was significantly different between the basiliximab and steroid groups for patients who met the Milan criteria (5-year OS: 88.9% vs. 57.4%; log-rank test, *P = *0.022) (Figure 3b). The 5-year OS was similar for patients treated with basiliximab or steroids who met UCSF criteria (5-year OS: 83.5% vs. 58.5%; log-rank test, *P = *0.079) (Figure 3c).

The Cox proportional hazard regression multivariate model that included therapy group, gender, age, transplant year, TNM tumor staging, and Milan criteria, after controlling for the other variables, found higher TNM staging was associated with higher mortality (Stage III+ vs. Stage I, adjusted HR = 3.08, 95% CI: 1.28–7.42; *P = *0.012) (Table 5). This analysis also found that patients meeting the Milan criteria had a lower mortality (meeting vs. not meeting, adjusted HR = 0.35, 95% CI: 0.17–0.73; *P = *0.005).

**Table 5:** Cox proportional hazard regression model for overall survival.

	Univariate		Multivariate†	
	crude HR (95% CI)	*P*-value	adjusted HR (95% CI)	*P*-value
Group				
Basiliximab	1.08 (0.68–1.72)	0.733	0.58 (0.27–1.21)	0.146
Steroid	1.00 (reference)	–	1.00 (reference)	–
Gender				
Female	1.00 (reference)	–	1.00 (reference)	–
Male	0.98 (0.52–1.87)	0.961	0.89 (0.46–1.72)	0.723
Age (y)				
<50	1.00 (reference)	–	1.00 (reference)	–
≥50	0.71 (0.45–1.12)	0.140	0.64 (0.40–1.02)	0.059
AFP^1^				
<200	1.00 (reference)	–		
≥200	1.54 (0.97–2.45)	0.067		
Transplant year				
2003–2005	0.86 (0.54–1.37)	0.516	0.57 (0.27–1.18)	0.130
2006–2009	1.00 (reference)	–	1.00 (reference)	–
Child–Pugh score^2^				
5–6	1.00 (reference)	–		
7–9	0.72 (0.44–1.17)	0.180		
10–15	0.91 (0.43–1.89)	0.792		
Diabetes mellitus				
No	1.00 (reference)	–		
Yes	0.94 (0.41–2.16)	0.879		
HBV				
No	1.00 (reference)	–		
Yes	0.47 (0.25–0.88)	0.019		
Cirrhosis				
No	1.00 (reference)	–		
Yes	0.44 (0.24–0.82)	0.010		
HCC				
Primary liver cancer	1.00 (reference)	–		
Recurrent hepatocellular carcinoma	1.38 (0.63–3.03)	0.420		
No. of tumor				
<2	1.00 (reference)	–		
≥2	1.29 (0.82–2.02)	0.278		
Diameter of largest tumor (cm)				
<5	1.00 (reference)	–		
≥5	2.35 (1.49–3.71)	0.0002		
TNM tumor staging for HCC, n (%)				
Stage I	1.00 (reference)	–	1.00 (reference)	–
Stage II	1.84 (0.85–4.01)	0.122	1.50 (0.67–3.38)	0.327
Stage III+	5.54 (2.69–11.42)	<0.0001	3.08 (1.28–7.42)	0.012
Milan Criteria^2^, n (%)				
Within Milan	0.21 (0.11–0.38)	<0.0001	0.35 (0.17–0.73)	0.005
Beyond Milan	1.00 (reference)	–	1.00 (reference)	–
UCSF Criteria^1^, n (%)				
Within UCSF	0.22 (0.13–0.38)	<0.0001		
Beyond UCSF	1.00 (reference)	–		
Preoperative antiviral therapy, n (%)				
No	1.00 (reference)	–		
Yes	1.14 (0.69–1.88)	0.616		

1 n = 173;

2 n = 177.

† In the multivariate model, data of 177 subjects were included.

AFP = alpha-fetoprotein; CI = confidence interval; HBV = hepatitis B virus; HCC = hepatocellular carcinoma; HCV = hepatitis C virus; HR = hazard ratio; UCSF = University of California San Francisco.

The Cox proportional hazard regression multivariate model for DFS that included therapy group, gender, age, transplant year, TNM tumor staging, and UCSF criteria, after controlling for the other variables, also found higher TNM staging was associated with higher rate of HCC recurrence (Stage III+ vs. Stage I, adjusted HR = 3.02, 95% CI: 1.35–6.78; *P = *0.007) (Table 6). This analysis also found that patients meeting the UCSF criteria had lower recurrence of HCC (within vs. beyond, adjusted HR = 0.37, 95% CI: 0.20–0.71; *P = *0.003).

**Table 6:** Cox proportional hazard regression model for disease-free survival.

	Univariate		Multivariate	
	crude HR (95% CI)	*P*-value	adjusted HR (95% CI)	*P*-value
Group				
Basiliximab	0.98 (0.65–1.47)	0.913	0.53 (0.27–1.06)	0.073
Steroid	1.00 (reference)	–	1.00 (reference)	–
Gender				
Female	1.00 (reference)	–	1.00 (reference)	–
Male	1.05 (0.58–1.89)		0.83 (0.46–1.51)	0.541
Age (y)				
<50	1.00 (reference)	–	1.00 (reference)	–
≥50	0.76 (0.51–1.13)		0.72 (0.48–1.09)	0.118
AFP^1^				
<200	1.00 (reference)	–		
≥200	1.64 (1.08–2.49)			
Transplant year				
2003–2005	0.98 (0.65–1.47)		0.57 (0.29–1.11)	0.098
2006–2009	1.00 (reference)	–	1.00 (reference)	–
Child–Pugh score^2^				
5–6	1.00 (reference)	–		
7–9	0.65 (0.42–1.01)			
10–15	0.90 (0.47–1.73)			
Diabetes mellitus				
No	1.00 (reference)	–		
Yes	1.33 (0.67–2.64)			
HBV				
No	1.00 (reference)	–		
Yes	0.50 (0.27–0.92)	0.025		
Cirrhosis				
No	1.00 (reference)	–		
Yes	0.47 (0.26–0.85)	0.012		
HCC				
Primary liver cancer	1.00 (reference)	–		
Recurrent hepatocellular carcinoma	1.07 (0.52–2.22)	0.855		
No. of tumor				
<2	1.00 (reference)	–		
≥2	1.30 (0.87–1.95)	0.201		
Diameter of largest tumor (cm)				
<5	1.00 (reference)	–		
≥5	2.57 (1.71–3.86)	<0.0001		
TNM tumor staging for HCC, n (%)				
Stage I	1.00 (reference)	–	1.00 (reference)	–
Stage II	1.72 (0.87–3.40)	0.118	1.56 (0.77–3.15)	0.219
Stage III+	5.47 (2.90–10.29)	<0.0001	3.02 (1.35–6.78)	0.007
Milan Criteria^2^, n (%)				
Within Milan	0.22 (0.13–0.38)	<0.0001		
Beyond Milan	1.00 (reference)	–		
UCSF Criteria^1^, n (%)				
Within UCSF	0.22 (0.13–0.36)	<0.0001	0.37 (0.20–0.71)	0.003
Beyond UCSF	1.00 (reference)	–	1.00 (reference)	–
Preoperative antiviral therapy, n (%)				
No	1.00 (reference)	–		
Yes	1.36 (0.88–2.10)	0.172		

1 n = 173;

2 n = 177.

† In the multivariate model, data of 173 subjects were included.

AFP = alpha-fetoprotein; HBV = hepatitis B virus; HCC = hepatocellular carcinoma; HCV = hepatitis C virus; UCSF, University of California San Francisco.

## Discussion

This study compared the efficacy and safety of immunosuppressive therapy based on either basiliximab or corticosteroids in Chinese HCC patients following liver transplantation. Although all patients received 1 dose of methylprednisone during the operation, the patients treated with basiliximab did not receive steroids during the post-operative period. Patients who received basiliximab had a significantly lower incidence of postoperative *de novo* diabetes and long-term *de novo* diabetes than patients who received steroids. The rates of *de novo* hypertension, *de novo* hyperlipidemia, acute rejection, and HCC recurrence were similar between the groups. The median OS and DFS, and the 5-year OS and DFS were comparable between the two groups. However for patients who met the Milan criteria, 5-year OS of patients treated with basiliximab was longer compared with those who received steroids.

The immune system plays a direct role in controlling the tumor growth, and evidence is accumulating that the choice of immunosuppressive therapy following HCC-related liver transplantation may affect treatment outcomes such as survival and HCC recurrence [21], [22]. For example, sirolimus (an inhibitor mTOR) based therapy is associated with longer recurrence-free survival, OS, and lower recurrence-related mortality than tacrolimus-based therapies [22], [25]–[27]. Several studies have indicated that steroid therapy may impact HCC recurrence following transplantation. One study found that a risk factor for HCC recurrence following transplantation was the dose of steroids given within 180 days of transplantation [28]. Another study found that basiliximab plus tacrolimus resulted in lower HCC recurrence than a tacrolimus-based treatment regimen that reduced steroid use over 3–6 months [29]. This same study found that removal of steroid therapy 3 months after transplantation was associated with a lower 1-year survival rate than steroid-maintenance therapy (39% vs. 69%; *P*<0.05) [29]. Our study did not find a difference in the HCC recurrence rate between treatments. This may be due to, at least in part, to differences in the patient criteria used for transplant eligibility, or different samples sizes. How certain immunosuppressive regimens influence HCC recurrence it not clear. Some findings suggest that steroids may result in protection of tumor cells from apoptosis [30]–[32]. Further studies are required to understand the underlying molecular mechanisms that influence how certain immunosuppressive regimens influence HCC recurrence in the transplant recipients.

Similar to our findings, prior studies have not found a difference in the OS rate, or HCV of HBV infection rates, between basiliximab and steroid containing treatments [16], [19]. In our study, there was difference in 5-year OS for patients meeting the Milan criteria who were treated with steroids compared with those receiving basiliximab (88.9% vs. 57.4%, respectively; log-rank test, *P = *0.022). These findings suggest that long-term steroid treatment can have a negative outcome for the subclass of patients that meet the Milan criteria. The reasons for the decrease in OS associated with steroid use in some patients are not clear, but may reflect the impact of steroid-associated adverse effects such a diabetes mellitus. Ours and prior studies [11], [12], [14] found the proportion of patients developing postoperative diabetes was lower (although not always significantly lower) in steroid-free compared with steroid-containing immunosuppressive regimens. Although multiple studies indicate the negative effects associated with steroid use in liver transplant patients, steroid-avoidance protocols are not generally implemented in most clinical settings due to the concern of acute rejection.

The effect of steroids on the rate of acute rejection is not clear; some studies have found that the presence of steroids in the immunosuppressive protocol was associated with higher acute graft rejection [12], [33], [34], while others, like this study, have not found this association [11], [13], [14].

Two prior studies have compared the efficacy and safety of basiliximab versus steroid-based immunosuppressive therapy [16], [19]. Similar to our findings, in one study basiliximab was associated with lower rates of diabetes than the steroid-containing therapy [19]. However, in the other study basiliximab and steroid therapies were similar in regards to the proportion of patients developing diabetes [16]. The differences in the results may reflect differences in the study populations, as the prior studies included other patients in addition to those with HCC. It may also result from differences in immunosuppressive regimens [16], [19]. The observation in our study that patients who met the Milan criteria and were treated with basiliximab had longer 5-year OS than those receiving steroids is consistent with patients meeting this criteria having a better prognosis [8].

In this study, a higher proportion of patients treated with basiliximab had postoperative infections, including intra-abdominal abscesses. This may reflect that basiliximab therapy requires the therapeutic target concentration of tacrolimus to be rapidly achieved, hence the overall initial dose of tacrolimus was higher in the basiliximab than the steroid group. The increased immunosuppression resulting from the high levels of tacrolimus may have promoted infections in patients prone to infections.

There are a number of limitations of this study that should be taken into consideration, which include the small number of patients in each group, relatively short follow-up length and the retrospective nature of the study. In addition, all patients who received a liver transplant prior to 2006 were given steroid therapy, and most patients from 2007 to 2009 received basiliximab. This non-random distribution may have possibly confounded some of the findings. However, there were no differences in operative or other treatment protocols between those two time periods. The high mortality rate may blind the real effect of the immunosuppression protocol on survival. Lastly, many Chinese patients carry HBV infection and more than 90% of the patients in this study had a history of HBV infection. In contrast, only about 1% had a history of HCV infection. Thus, a comparison of underlying disease (HBV negative and HCV positive) with respect to the protocols cannot be performed. However, a recent study indicated that survival outcomes after liver transplantation were significantly better in HBV-HCC patients than in HCV-HCC patients [35].

## Conclusion

This study found that the use of basiliximab instead of steroids as part of the immunosuppression therapy following liver transplantation in HCC patients was associated with a longer 5-year overall survival in patients that met the Milan criteria and a lower occurrence of diabetes. There was no difference between treatments in regards to HCC recurrence. These findings are consistent with the negative impact of steroids on morbidity and mortality and suggest that basiliximab is an effective immunosuppression therapy following liver transplantation.
